# Identification of Nine mRNA Signatures for Sepsis Using Random Forest

**DOI:** 10.1155/2022/5650024

**Published:** 2022-03-19

**Authors:** Jing Zhou, Siqing Dong, Ping Wang, Xi Su, Liang Cheng

**Affiliations:** ^1^Intensive Care Unit, The Second Affiliated Hospital of Harbin Medical University, Harbin 150081, China; ^2^Genomics Research Center, Harbin Medical University, Harbin 150081, China; ^3^Beidahuang Industry Group General Hospital, Harbin 150001, China; ^4^College of Bioinformatics Science and Technology, Harbin Medical University, Harbin 150081, China; ^5^Foshan Maternity & Child Healthcare Hospital, Southern Medical University, Foshan 528000, China

## Abstract

Sepsis has high fatality rates. Early diagnosis could increase its curating rates. There were no reliable molecular biomarkers to distinguish between infected and uninfected patients currently, which limit the treatment of sepsis. To this end, we analyzed gene expression datasets from the GEO database to identify its mRNA signature. First, two gene expression datasets (GSE154918 and GSE131761) were downloaded to identify the differentially expressed genes (DEGs) using Limma package. Totally 384 common DEGs were found in three contrast groups. We found that as the condition worsens, more genes were under disorder condition. Then, random forest model was performed with expression matrix of all genes as feature and disease state as label. After which 279 genes were left. We further analyzed the functions of 279 important DEGs, and their potential biological roles mainly focused on neutrophil threshing, neutrophil activation involved in immune response, neutrophil-mediated immunity, RAGE receptor binding, long-chain fatty acid binding, specific granule, tertiary granule, and secretory granule lumen. Finally, the top nine mRNAs (MCEMP1, PSTPIP2, CD177, GCA, NDUFAF1, CLIC1, UFD1, SEPT9, and UBE2A) associated with sepsis were considered as signatures for distinguishing between sepsis and healthy controls. Based on 5-fold cross-validation and leave-one-out cross-validation, the nine mRNA signature showed very high AUC.

## 1. Introduction

As a clinical syndrome, sepsis has been accompanied by human society from ancient times to the present [1]. Sepsis and septic shock have high fatality rates and consume a large amount of medical resources. Since the launch of save sepsis in the early 2000s, the treatment outcomes of patients with sepsis have improved. But the case fatality rate for sepsis remains at 25 to 30 percent, and when shock occurs, it can be as high as 40 to 50 percent [2]. After decades of research, there is still no specific treatment for sepsis. The improvement in patient outcomes came primarily from nonspecific interventions, including fluid resuscitation, early application of antibiotics, and elimination of the source of infection ([3] #5; [4] #8478; [5] #8582; [6] #49). An important reason for this disheartening situation is that the definitions of sepsis and septic shock cover a very heterogeneous population of patients. The causes are so varied that it is difficult to find a common treatment for these conditions.

How to classify patients with sepsis is one of the key areas of research on sepsis and other diseases [7–9], though biomarkers have been the subject of intensive research for decades ([10] #71; [11] #15; [12] #8853; [13] #431; [14] #673; [15] #50). For example, procalcitonin has been included in treatment guidelines [16], but there is currently no reliable biomarker to distinguish between infected and uninfected patients. Only 30-40% of patients with sepsis or septic shock have positive blood cultures. New technologies such as high-throughput technologies (genomics, transcriptomics, etc.) have been used to better identify subsets of patients with sepsis, to identify patients at high risk of developing sepsis, and to provide the possibility for rapid and accurate diagnosis of infection [17, 18, 19].

This study analyzed microarray dataset from public gene expression database, to obtain differentially expressed genes (DEGs) between sepsis and healthy people, and then, a random forest model was performed on the DEGs to select more import biomarkers. Next, we performed gene functional enrichment analysis on the DEGs selected to analyze the function module of the DEGs and to uncover how the DEGs contribute to sepsis. Our study aims to detect neglected biomarkers of sepsis to better distinguish between sepsis patients and healthy controls.

## 2. Materials and Methods

### 2.1. Data Resource

To identify potential gene signatures associated with sepsis, we got two gene expression datasets (GSE154918 and GSE131761) [20, 21] from the GEO database (https://www.ncbi.nlm.nih.gov/geo/), GSE154918 dataset as primary research data and GES131761 as supplementary data.

Totally, 109 samples from GSE154918 dataset were collected from 19 septic shock patients, 20 sepsis patients, 12 uncomplicated infection patients, and 40 healthy volunteers. Supplementary validation dataset GSE131761 was collected from 81 septic shock patients and 15 healthy volunteers. All samples were collected from peripheral blood. The diagnosis of septic shock was according to the Sepsis 3.0 criteria [3].

### 2.2. Identification of DEGs

The workflow is shown in Figure 1. DEGs were calculated between sepsis samples (uncomplicated infection, sepsis, and septic shock) and healthy control using Limma package [22] with *p* value < 0.05 and ∣*logFC* | >1 as threshold.

### 2.3. Random Forest Model

Random forest model was performed using Python machine learning library Scikit-learn [23], with expression matrix of all genes as feature and disease state as label as other researches [1]. We set 1000 random forest trees and operated 5-fold cross-validation and leave-one-out cross-validation to evaluate the performance of the model. Feature importance was collected from the random forest model after training and assessment, and then, we sorted the features by feature importance and chose top *n* features to reconstruct random forest, accessing the best combination of gene signatures [24].

### 2.4. Functional and Pathway Enrichment Analyses

Gene enrichment analysis of DEGs was based on Gene Ontology (GO) database from molecular function, cellular component, and biological process using R package ClusterProfiler [25]; pathways with adjusted *p* value < 0.05 were selected as significant enriched pathways [26].

## 3. Results

### 3.1. Identification of DEGs

Gene expression difference was calculated between three sepsis groups and healthy control, respectively. 530 differentially expressed genes (DEGs) were found in uncomplicated infection patients compared with healthy control, 727 DEGs were found in sepsis samples, 1414 DEGs were found in sepsis shock samples, and 384 common DEGs were found in the above three contrast groups (Figure 2). We found that as the condition worsens, more genes were under disorder condition.

### 3.2. Features Selected by Random Forest

Next, we performed random forest [15, 27] to select important genes of the DEGs of the above three contrast groups, with gene expression matrix of DEGs as feature and health state as label; we selected the genes with feature *importance* > 0 as the most important genes. We, respectively, found 440, 657, and 1018 DEGs in uncomplicated infection vs. healthy control, sepsis vs. healthy control, and sepsis shock vs. healthy control, and 279 genes were common among the three (Figure 3).

### 3.3. Enrichment Analysis of Intersection Important DEGs

We further performed functional analyses for 279 important DEGs to explore the underlying biological roles. Multiple GO-BP terms were associated with neutrophil degranulation, neutrophil activation involved in immune response, and neutrophil-mediated immunity. The DEGs played essential roles in GO-MF terms containing 2 more enriched terms: RAGE receptor binding and long-chain fatty acid binding. The GO-CC revealed that these DEGs were mainly enriched in specific granule, tertiary granule, and secretory granule lumen (Figure 4).

### 3.4. Biomarkers Distinguishing Disease States

To detect biomarkers to distinguish three disease-state patients and healthy patients, we further performed random forest on three disease states and healthy samples together, sorted the feature importance, and selected the top *n* (1-50) gene features to reconstruct random forest model to access the best biomarker combination. We found that when 6 features were selected, the accuracy of the model reached 0.895, and the accuracy of model began to decline since more than 9 features were selected. Therefore, the first 9 characteristics were selected as potential biomarkers to predict different sepsis states (Figure 5).

### 3.5. Supplement Validation

In order to assess the availability of the 9 biomarkers, we used a supplementary validation dataset to build random forest model using these 9 biomarkers as feature. Since the biomarker MCEMP1 was not sequenced because of lacking probe, only 8 biomarkers were sequenced in supplement dataset, so we only evaluated the 8 biomarkers. We found that the model performed good to distinguish sepsis from healthy control in supplement dataset. Then, we further calculated the gene expression difference between sepsis and healthy control samples in supplement dataset, and we found that 6 out of 8 biomarkers were DEGs in supplement dataset (Table 1).

## 4. Discussion

According to the Sepsis 3.0 definition, sepsis is a life-threatening organ dysfunction resulting from an infection-induced host response disorder. Neutrophils are the main immune-cell barrier against pathogens, but they can be a double-edged sword in sepsis because they play a role in both proinflammatory response and anti-inflammatory response. We hypothesize that the immune signature of sepsis can be determined early by the phenotype of neutrophils and distinguish sepsis from noninfectious inflammatory syndromes. It is important to screen for features that are considered important in the biology of sepsis but alone are not distinguishable to clearly distinguish sepsis. Sepsis is thought to be an immune imbalance in which pathogens evade the host's defense mechanisms and continue to stimulate and destroy host cells. Many of the protective immune mechanisms activated early in the disease become harmful and are associated with excessive inflammation and immunosuppression. The host response of sepsis involves the coexistence of inflammatory and anti-inflammatory responses, involving different organs, systems, and cell types [28].

We conducted a differential analysis of data from a group of three sepsis severity levels and healthy controls and found that the number of differential genes in sepsis patients increased according to the severity of the disease, suggesting that more genes became dysregulated with the severity of the disease. There were 279 differentially expressed genes in all three kinds of severe infection, which may play roles in the onset and progression of sepsis. Functional enrichment analysis showed that biological processes were most significantly enriched in neutrophil activation, immune activation, inflammatory response, and bacterial response.

In GO-MF analysis, DEGs were significantly enriched in RAGE receptor binding and long-chain fatty acid binding. A meta-analysis showed that RAGE inhibition had a significant advantage in multiple microbial infections. For G^+^ bacterial infection, RAGE suppression reduced bacterial growth and transmission, inflammatory cell flow, plasma cytokine levels, and lung damage. This paper concluded that RAGE inhibition had beneficial effects on the outcomes of animal models of sepsis with different causes [29]. There are few studies on long-chain fatty acid binding and sepsis. This article is one of them. Extraenteral pathogenic E. coli can cause diseases such as urinary tract infections and sepsis. Mucus is the main nutrient source of Escherichia coli in the intestinal tract, and genes directly or indirectly related to the fatty acid oxidation pathway contribute to the adaptation and migration of ExPEC [30].

In our study, the remarkable GO-CC terms are associated with neutrophil degranulation, such as tertiary granule, specific granule, and secretory granule lumen. Neutrophils are one of the most important cells in the host's natural defense. The following are the granules in neutrophil cytoplasm: azurophilic granule, specific granules, gelatinase granules, and secretory vesicles. They all play very important roles. Neutrophil dysregulation is present in sepsis. Many evidence suggest that neutrophil threshing molecules are of value in the diagnosis and prognosis of sepsis. Monitoring neutrophil function may help identify early sepsis [31].

We used the random forest to select 9 characteristic genes as potential biomarkers for predicting sepsis: MCEMP1, PSTPIP2, CD177, GCA, NDUFAF1, CLIC1, UFD1, SEPT9, and UBE2A. Some of these genes have been confirmed in experiments or have also been widely concerned in bioinformatics studies.

MCEMP1 is involved in the regulation of mast cell differentiation or innate immune response. In our study, MCEMP1 gene expression was increased in sepsis. Chen et al. [32]. established a cecal ligation and puncture-induced sepsis mouse model to determine the expression of mast cell expression membrane protein 1 (MCEMP1). They observed that MCEMP1 was highly expressed in septic mice. Loss of MCEMP1 can promote T lymphocyte and NK cell activity, increase immunoglobulin expression, inhibit the release of inflammatory factors, and reduce T lymphocyte apoptosis. They also found that downregulation of lncRNA NEAT1 could inhibit MCEMP1, thereby promoting the immunosuppression effect of Mir-125 on sepsis mice. This may be a potential therapeutic target for sepsis. Xie et al. found that MALAT1 upregulates MCEMP1 by binding to Mir-23a, thereby promoting inflammatory response in sepsis mice [33].

Proline-serine-threonine-phosphatase-interacting protein 2 (PSTPIP2) belongs to the F-BAR family of proteins and is mainly expressed in macrophages. In recent years, PSTPIP2 has been found to play an important role in congenital immune diseases and acquired immune diseases (AIDS) [34]. Chen et al. [35] studied biomarkers of Escherichia coli-induced sepsis. They analyzed 4 microarray datasets from GEO database and identified 54 DEGs. Eight different genes were found between sepsis patients and controls. Furthermore, differential expression of the candidate gene was verified by human blood model in vitro. qPCR results suggested that PSTPIP2 may be closely related to Escherichia coli-induced sepsis.

Neutrophils play an important role in the pathophysiology of sepsis and are the primary defense against infection. A transcriptome study was performed on purified neutrophils from patients with septic shock to identify genes that were differentially expressed during the first week of illness compared with healthy controls. The results were confirmed at the protein level. They found that 364 differentially expressed genes were upregulated and 328 downregulated in patients with sepsis. CD177mRNA showed the most significant difference between patients and healthy controls. This is consistent with our findings, which also found that CD177 was significantly upregulated in sepsis patients [36].

Yang and Li [37] applied bioinformatics to study the molecular mechanism of sepsis. Transcriptome data (GSE12624) were downloaded from Gene Expression Omnibus database for protein-protein interaction network analysis. Twenty-four differentially expressed clusters were identified by ANCOVA global test, including 12 clusters in sepsis samples and 12 clusters in nonsepsis samples. 207 biomarker genes were extracted from the first 6 clusters by SVM method, and 10 genes including GCA were considered as potential biomarkers.

Tang et al. [38] explored the relationship between septic shock and AKI by analyzing codifferentially expressed genes (co-DEGs) in the hope of identifying possible genetic markers for septic shock-associated AKI. They downloaded two gene expression datasets (GSE30718 and GSE57065). DEGs related to septic shock and AKI were searched to clarify the molecular mechanism of DEGs through function analysis (GO), pathway enrichment analysis (KEGG), and protein interaction (PPI) network analysis. They also assessed co-DEGs and corresponding predictive miRNAs associated with septic shock and AKI. 16 genes, including NDUFAF1, were found to be involved in septic shock-associated AKI. Our study also found that NDUFAF1 expression was upregulated in patients with sepsis.

UBE2A, also called HHR6A or UBC2, can be expressed in a variety of tissues. Current studies mainly focus on cognitive impairment and skeletal muscle metabolism, but we have not found reports that UBE2A is directly related to sepsis. UBE2A may be associated with increased skeletal muscle protein catabolic activity in a number of diseases and malnutrition states, such as cancer, sepsis, and diabetes. Sepsis is often accompanied by septic encephalopathy, which is mainly manifested by changes in cognitive function and state of consciousness. It is necessary to further study whether UBE2A expression is abnormal in patients with septic encephalopathy [39, 40].

In our study, there were 9 major differential genes involved in the development of sepsis. Five of these genes have been reported, indicating that the biomarkers selected by our random forest model have high diagnostic value. CLIC1, UFD1, SEPT9, and UBE2A are new biomarkers found by us through the random forest model, and there is no research report related to sepsis so far. These four genes may serve as relevant targets for the diagnosis and treatment of sepsis. Future in vitro and in vivo studies are needed to analyze the functions and pathways of these genes in the pathophysiology of sepsis. Further studies in more sepsis patients are needed to confirm the diagnostic value of the selected genes.

## 5. Conclusions

In this study, bioinformatics methods were used to analyze two septic shock-related datasets (GSE154918 and GES131761) and identify differentially expressed genes (DEGs) from GEO. We found that the number of differentially expressed genes increased with the increase of sepsis severity. It indicates that there are more genetic disorders from sepsis to septic shock. GO gene enrichment analysis showed that differential gene expression was significantly enriched in neutrophil activation and degranulation pathways. RAGE pathway has been found to be closely related to the occurrence of sepsis. Nine genes, including MCEMP1, PSTPIP2, CD177, GCA, NDUFAF1, CLIC1, UFD1, SEPT9, and UBE2A, were identified to be associated with sepsis. Further studies of the role of these pathways and genes in sepsis patients or experiments are needed.

## Figures and Tables

**Figure 1:** The workflow of identifying molecular signature of sepsis. Gene different expression analysis was firstly performed on gene expression data, and then, random forest model was performed with expression of DEGs as feature. Next, the function of selected important DEGs from random forest was analyzed.

**Figure 2:** DEG numbers of the three contrast groups. The Venn diagram displays the DEG numbers of three contrast groups Inf1_P vs. healthy, Sepsis_P vs. healthy, and Shock_P vs. healthy.

**Figure 3:** Gene feature numbers of the three contrast groups after performing random forest. The Venn diagram displays the gene feature numbers of the three contrast groups Inf1_P vs. healthy, Sepsis_P vs. healthy, and Shock_P vs. healthy.

**Figure 4:** Gene enrichment result of 279 important features. Based on Gene Ontology database, from molecular function, cellular component, and biological process, respectively (*p* < 0.05).

**Figure 5:** Relationship between the selected top feature number and model evaluation score. The line chart shows that the random forest evaluation score changes with the increase of feature number.

**Table 1:** DEG analysis in supplement dataset of 9 biomarkers. MCEMP1 was not sequenced in supplement dataset.

Biomarkers	logFC	Adj. *p* values
CLIC1	1.063383	2.56E-17
MCEMP1	—	—
PSTPIP2	1.257539	2.26E-12
UFD1	0.627806	3.35E-12
CD177	4.637112	9.32E-23
SEPT9	-1.2021	2.32E-22
NDUFAF1	1.206761	6.17E-16
GCA	1.582514	6.45E-16
UBE2A	0.595547	1.55E-12

## Data Availability

The data used to support the findings of this study have been deposited in the GEO database repository (GSE154918 and GES131761).
